The article "Disruption of embryonic ROCK signaling reproduces the sarcomeric phenotype of hypertrophic cardiomyopathy" was retracted in 2020. Reason: fabricated or falsified data.

# Disruption of embryonic ROCK signaling reproduces the sarcomeric phenotype of hypertrophic cardiomyopathy

**DOI:** 10.1172/jci.insight.125172

**Published:** 2019-04-18

**Authors:** Kate E. Bailey, Guy A. MacGowan, Simon Tual-Chalot, Lauren Phillips, Timothy J. Mohun, Deborah J. Henderson, Helen M. Arthur, Simon D. Bamforth, Helen M. Phillips

**Affiliations:** 1 Institute of Genetic Medicine, Newcastle University, Newcastle upon Tyne, United Kingdom.; 2 The Francis Crick Institute, London, United Kingdom.

**Keywords:** Cardiology, Cardiovascular disease

## Abstract

Sarcomeric disarray is a hallmark of gene mutations in patients with hypertrophic cardiomyopathy (HCM). However, it is unknown when detrimental sarcomeric changes first occur and whether they originate in the developing embryonic heart. Furthermore, Rho kinase (ROCK) is a serine/threonine protein kinase that is critical for regulating the function of several sarcomeric proteins, and therefore, our aim was to determine whether disruption of ROCK signaling during the earliest stages of heart development would disrupt the integrity of sarcomeres, altering heart development and function. Using a mouse model in which the function of ROCK is specifically disrupted in embryonic cardiomyocytes, we demonstrate a progressive cardiomyopathy that first appeared as sarcomeric disarray during cardiogenesis. This led to abnormalities in the structure of the embryonic ventricular wall and compensatory cardiomyocyte hypertrophy during fetal development. This sarcomeric disruption and hypertrophy persisted throughout adult life, triggering left ventricular concentric hypertrophy with systolic dysfunction, and reactivation of fetal gene expression and cardiac fibrosis, all typical features of HCM. Taken together, our findings establish a mechanism for the developmental origin of the sarcomeric phenotype of HCM and suggest that variants in the *ROCK* genes or disruption of ROCK signaling could, in part, contribute to its pathogenesis.

## Abstract 2

Disruption of ROCK activity in embryonic cardiomyocytes revealed a developmental origin for hypertrophic cardiomyopathy.

## Introduction

Familial hypertrophic cardiomyopathy (HCM) is often referred to as a disease of the sarcomere, as a large number of mutations have been found in sarcomere-related genes (1). However, the mutations identified so far only account for ~50% of familial HCM cases (2), suggesting more candidate genes remain to be discovered. Furthermore, although there are numerous transgenic mouse models of HCM, few of the published studies have followed the structural impact of HCM mutations on the sarcomeres prior to initiation of cardiac dysfunction in the adult. For instance, deleterious events unique to the embryonic heart may have lasting impact on the function of the adult myocardium. Moreover, identification of further genetic variants associated with HCM and greater understanding of disease progression will help in understanding the variability in HCM disease and penetrance.

The article "Disruption of embryonic ROCK signaling reproduces the sarcomeric phenotype of hypertrophic cardiomyopathy" was retracted in 2020. Reason: fabricated or falsified data.

Rho kinase (ROCK) is a serine/threonine protein kinase that is critical for regulating phosphorylation of several sarcomeric proteins — myosin light chain 2 (Mlc2) (3), cardiac troponin I (cTnI), and cardiac Troponin T (cTnT) (4) — that all have important roles in regulating sarcomeric structure. There are 2 isoforms, ROCK1 and ROCK2, and they are the main downstream effectors of the small Rho GTPase RhoA. The active form of RhoA, GTP-RhoA, binds to the Rho-binding domain of ROCK and hence can activate both of these proteins. In addition to sarcomeric proteins, many proteins are phosphorylated by ROCK such that it is involved in a number of diverse cellular activities, including actin cytoskeleton organization and muscle contraction (5), that are critical properties of cardiomyocyte function. Therefore, as HCM mutations are believed to affect the efficiency of sarcomere assembly (6) or cause sarcomere dysfunction including altered contractility (7), we hypothesized that the 2 ROCK isoforms would be ideal potential candidate genes for HCM if their function were found to be disrupted in cardiomyocytes.

Both isoforms of ROCK are expressed in the developing heart from the cardiac crescent stage at E7.5 (8, 9) and are required for migration of cardiac precursor cells (8). Although *ROCK1*- or *ROCK2*-null mice have been reported to be embryonic lethal, viability is influenced by genetic background (10–12). The role of ROCK in cardiac hypertrophy and heart failure has previously been studied in adult mouse transgenic models with pathological-induced conditions, such as pressure overload–induced cardiac hypertrophy in the heart. Mouse models have implicated ROCK1 in the pathogenesis of cardiac fibrosis (12) and the transition from cardiac hypertrophy to heart failure (13), and ROCK2 in regulating cardiac hypertrophy (14), in response to cardiac-targeted pathological-induced stimuli to induce cardiac hypertrophy. However, to our knowledge no studies to date have specifically focused on the endogenous role of ROCK in embryonic cardiomyocytes in the absence of any additional disease factors. Here we used the well-established *ROCKDN* mouse model (15) to target ROCK function in embryonic cardiomyocytes, using the same rationale as in our previous work (16, 17), and tracked the long-term effect on cardiomyocyte function in the adult heart. Hence, we were able to study disease progression from initial onset during embryology to overt disease pathology associated with altered cardiac function. *ROCKDN* encodes a dominant negative ROCK protein that disrupts endogenous ROCK activity and is conditionally expressed in cells expressing Cre recombinase. We identified a mechanism in *ROCKDN^Gata5-Cre^* mutant mice, where there was disruption of the sarcomeres in embryonic cardiomyocytes, alongside reduced phosphorylation of troponins and reduced cardiomyocyte proliferation. This led to delayed maturation and development of the ventricular wall, and compensatory hypertrophy of fetal cardiomyocytes. The sarcomeric disruption and hypertrophy persisted into adulthood, subsequently transitioning to left ventricular (LV) dysfunction, emulating many of the clinical and histological features of HCM. Therefore, this transgenic mouse models the sarcomeric phenotype of HCM where the transient developmental downregulation of ROCK led to HCM in adult life, highlighting that HCM can have a developmental origin, which is clinically unidentifiable until the presentation of the disease.

The article "Disruption of embryonic ROCK signaling reproduces the sarcomeric phenotype of hypertrophic cardiomyopathy" was retracted in 2020. Reason: fabricated or falsified data.

## Results

### Early downregulation of ROCK function in cardiomyocytes led to defects in embryonic ventricular wall development.

To evaluate *ROCK* expression in the embryonic heart, we used RNAscope probes specific for *ROCK1* and *ROCK2*, and showed that both isoforms were expressed uniformly in cardiomyocytes throughout the ventricular wall at E9.5 and E10.5 (Supplemental Figure 1, A–H; supplemental material available online with this article; https://doi.org/10.1172/jci.insight.125172DS1). Therefore, to investigate the function of ROCK specifically within developing cardiomyocytes, we used the *ROCKDN* transgenic mouse model (15–21), bred with either *TnT-Cre* (22) or *Gata5-Cre* (23) transgenic mice and with *WT1-ERT-Cre* (24) transgenic mice to target ROCK function in the epicardium. Expression of *ROCKDN* and removal of the CAT box only in the presence of *Cre* expression for each mouse cross were confirmed by quantitative real-time PCR (qRT-PCR) (Supplemental Figure 1, I–L).

In addition, the *R262ReYFP* reporter line (25) was used to track cells with *Cre* activity and confirmed uniform expression of *TnT-Cre* throughout cardiomyocytes at E10.5 (Supplemental Figure 2, A–D, and Supplemental Table 1A). 131 *ROCKDN^TnT-Cre^* mutant embryos were collected from E9.5 to E17.5 (Supplemental Table 2A), and no mutant pups were collected from P0 onward. The is the first report to our knowledge to show that targeted disruption of ROCK activity in embryonic cardiomyocytes causes embryonic lethality. The phenotypes of the embryonic hearts were then examined by histology. In comparison to the control embryos, there were no obvious phenotypic differences in the development of the ventricular wall at E10.5 in *ROCKDN^TnT-Cre^* mutant embryos (Figure 1, E and M). However, from E11.5, the ventricular wall of the *ROCKDN^TnT-Cre^* mutant was visibly thinner, with fewer trabeculae compared with the control embryo (Figure 1, F and M). Measurements of the thickness of the compact myocardium at E10.5–E15.5 showed that the compact myocardial wall from E12.5 in *ROCKDN^TnT-Cre^* embryos was significantly thinner, and remained significantly thinner at E14.5 and E15.5 (Figure 1M). By E15.5, all the *ROCKDN^TnT-Cre^* hearts were dilated, with thin ventricular walls, no defined interventricular sulcus, and underdeveloped trabeculae (Figure 1, G and H). Externally, from E12.5, 12% of *ROCKDN^TnT-Cre^* embryos had edema, and by E15.5 this had increased to 23%, indicating inadequate cardiac function and possible heart failure (data not shown). This analysis showed that ROCK function is required in the embryonic cardiomyocytes for normal maturation and function of the ventricular wall from E11.5.

The article "Disruption of embryonic ROCK signaling reproduces the sarcomeric phenotype of hypertrophic cardiomyopathy" was retracted in 2020. Reason: fabricated or falsified data.

We speculated that the *ROCKDN^Gata5-Cre^* mutants might have a milder viable phenotype compared with the *ROCKDN^TnT-Cre^* mutants, hence allowing investigation of the impact of embryonic ROCK downregulation on the adult heart. This is because *Gata5-Cre* is expressed from E9.25 in a proportion of the cardiomyocytes. At E9.5, *Cre* expression was seen in 13% of cardiomyocytes in the right ventricle and 19% in the left ventricle (Supplemental Figure 2, E–H), rising to 55% and 68%, respectively, by E15.5 (Supplemental Table 1B). Furthermore, we would have the benefit of mosaicism, which allows cardiomyocytes in which ROCK function is disrupted to be directly compared with genetically unaffected cardiomyocytes within the same heart. However, *Gata5-Cre* is also expressed in the epicardium from E9.25 (23). As we wanted to discriminate the cardiomyocyte-specific function from any indirect epicardial role, we first confirmed that loss of ROCK activity in the epicardium did not affect the myocardium. *Cre* expression was activated at E9.5 in *ROCKDN^WT1-ERT-Cre^* litters, and the embryos were collected at E15.5. Cre expression was confirmed in the epicardium and epicardial derived cells (Supplemental Figure 2, M and N). However, no heart defects and in particular no ventricular wall defects were identified in any of the *ROCKDN^WT1-ERT-Cre^* mutant embryos (Supplemental Figure 2, O and P). Thus, ROCK function in the epicardium was not essential for ventricular wall maturation at this stage of development, and any heart defects identified in the *ROCKDN^Gata5-Cre^* mutants were due to the *Cre* expression in the cardiomyocytes of the ventricular wall.

The article "Disruption of embryonic ROCK signaling reproduces the sarcomeric phenotype of hypertrophic cardiomyopathy" was retracted in 2020. Reason: fabricated or falsified data.

*ROCKDN^Gata5-Cre^* mutants and control littermates were collected from E9.5 to adulthood: 380 mutant embryos, 67 mutant postnatal pups up to 1 month, and 38 mutant adults aged 2–16 months. At each age, the proportions of *ROCKDN^Gata5-Cre^* mutants were all within the expected Mendelian ratios, and there were no sudden deaths (Supplemental Table 2B), showing that *ROCKDN^Gata5-Cre^* mutants survived embryogenesis and developed into adult mice.

Expression analysis of hearts from *ROCKDN^Gata5-Cre^* mutants and control littermates showed that *ROCKDN* was strongly expressed in the mutants until P21, with a significant drop in expression levels between each time point until 3 months (Supplemental Figure 3A). Therefore, any defects seen in the adult hearts were not due to disruption of ROCK signaling in adulthood. No change in *Cre* expression or endogenous *ROCK1* and *ROCK2* expression was seen between control and mutant hearts in embryos or adults (Supplemental Figure 3, B–D).

Examination of the embryos by histology revealed that at E10.5, hearts from *ROCKDN^Gata5-Cre^* mutants were comparable to those from control littermates (Figure 1, A and I). However, there was visible thinning of the ventricular wall throughout the heart beginning at E11.5, which was very similar to the *ROCKDN^TnT-Cre^* mutants at the same age (Figure 1, F and G), and also evident at E14.5 and E15.5 (Figure 1, K, L, and N). Further detailed analysis of the LV and right ventricular (RV) walls, individually, showed that in control embryos from E15.5 the compact myocardial wall thickened steadily up to P21, with no significant difference in cell size between E15.5 and E16.5 (blue lines, Figure 2, A and B). In comparison, the thickness of the compact myocardium of the *ROCKDN^Gata5-Cre^* mutants increased significantly between E15.5 and E16.5 in both ventricles (red lines, Figure 2, A and B). However, in comparison to control hearts, from E16.5, there was a trend for the LV and RV walls in the *ROCKDN^Gata5-Cre^* mutants to remain thinner, and they were significantly thinner in both ventricles at P7 and P21. At E15.5, the *ROCKDN^Gata5-Cre^* mutant hearts had persisting immature trabeculae that were more pronounced than those in the control hearts, forming myocardial crypts, which are discrete clefts in the compact myocardium (Figure 2, C–F). These myocardial crypts remained more prevalent in the *ROCKDN^Gata5-Cre^* mutants in postnatal hearts (Figure 2, G–J), as no crypts were seen in control hearts. All of these structural phenotypic differences in the ventricular wall were identified in all of the *ROCKDN^Gata5-Cre^* mutants examined at each age. To confirm that the *ROCKDN^Gata5-Cre^* mutants did not have a noncompaction phenotype (highly trabeculated myocardium with prominent deep intertrabecular recesses), we used an established method to measure trabecular complexity (26). No significant increase in trabecular complexity was observed in *ROCKDN^Gata5-Cre^* fetal or postnatal mutant hearts compared with control hearts (Figure 2K). Thus, the results confirmed that these mice had a delay in maturation of the ventricular wall in *ROCKDN^Gata5-Cre^* mutants, as the compact myocardium failed to thicken and some trabeculae did not compact fully.

The article "Disruption of embryonic ROCK signaling reproduces the sarcomeric phenotype of hypertrophic cardiomyopathy" was retracted in 2020. Reason: fabricated or falsified data.

### Disruption of ROCK signaling leads to a delay in maturation of the ventricular wall.

As chemical inhibition of ROCK during mouse embryo culture had previously shown a decrease in proliferation in the whole heart (9), we speculated that the cause of the thin myocardium in the *ROCKDN^Gata5-Cre^* mutants was due to reduced cardiomyocyte proliferation and/or increased apoptosis. Therefore, we examined these processes in embryonic hearts at E10.5 and E11.5, coinciding with the first visual appearance of an abnormal ventricular wall in the *ROCKDN^Gata5-Cre^* mutants at E11.5. No significant difference in proliferation was seen at E10.5; however, there was a significant decrease in proliferation specifically in Cre-activated cardiomyocytes in the compact myocardium of both ventricles at E11.5 in the *ROCKDN^Gata5-Cre^* mutants (Figure 3, A–C). There was no change in Cre-negative proliferating cardiomyocytes and no difference in cell death using caspase-3 antibody staining (data not shown). Thus, the decrease in proliferation at E11.5 accounted for the subsequent thinning of the compact myocardium.

To explain the significant increase in compact wall thickness between E15.5 and E16.5 in *ROCKDN^Gata5-Cre^* mutants (Figure 2, A and B), we first hypothesized that there may be a “catch-up” acceleration in proliferation between these two ages. However, no significant differences in the percentage of all proliferating cardiomyocytes in the compact myocardium of the LV or RV was detected at either age (Figure 3D). Furthermore, cell counts from the compact myocardium showed that the average number of cardiomyocytes per field of view was significantly smaller throughout the heart at E16.5 and E17.5 in *ROCKDN^Gata5-Cre^* mutants (Figure 3E). The increase in thickness between E15.5 and E16.5 in *ROCKDN^Gata5-Cre^* mutants might therefore be due to an increase in cardiomyocyte hypertrophy.

At E16.5, cardiomyocytes were, on average, significantly larger (16% and 12%) in the LV and RV, respectively, in *ROCKDN^Gata5-Cre^* mutants compared with control cardiomyocytes (Figure 3, F, G, K, and L, and Supplemental Table 3A). This increase in hypertrophy was seen in both Cre-activated (green) and Cre-negative cardiomyocytes (unstained) (Figure 3, H–J), suggesting that all the cardiomyocytes were undergoing compensatory hypertrophy in order to maintain adequate cardiac function. In subsequent postnatal stages (up to P21), all of the cardiomyocytes remained significantly hypertrophic in the *ROCKDN^Gata5-Cre^* mutants compared with the controls (Figure 3, K and L).

The article "Disruption of embryonic ROCK signaling reproduces the sarcomeric phenotype of hypertrophic cardiomyopathy" was retracted in 2020. Reason: fabricated or falsified data.

Markers of cardiomyocyte maturity were examined to establish whether this process was delayed in the *ROCKDN^Gata5-Cre^* mutants. In agreement with published data (27), in control hearts, α–smooth muscle actin (α-SMA) was restricted to the compact myocardium by E15.5 and to smooth muscle of the coronary arteries by P4 (Figure 4, A–E). In *ROCKDN^Gata5-Cre^* mutants, however, α-SMA was still expressed in trabeculae at E15.5 and E17.5 (Figure 4, F, G, and K), and patchy staining throughout the ventricular wall was still evident at P7 (Figure 4J). Thus, disruption of ROCK function leads to a delay in the maturation of the cardiomyocytes. Therefore, embryonic cardiomyocytes require ROCK function for normal development and maturation of trabeculae and compact myocardium from E11.5.

### Reduced ROCK signaling causes disruption of sarcomeres in cardiomyocytes from E10.5 in ROCKDN^Gata5-Cre^ and ROCKDN^TnT-Cre^ mutants.

Having established that in both *ROCKDN^Gata5-Cre^* and *ROCKDN^TnT-Cre^* mutants a defect in the structure of the ventricular wall is first visible from E11.5, we then looked a day earlier at E10.5 to establish what intracellular abnormalities may have led to the abnormal wall development. We first looked at the integrity of sarcomeres in the *ROCKDN^Gata5-Cre^* mutants. At E9.25, when Gata5-Cre was first expressed, the expression pattern of cTnI was identical in control and *ROCKDN^Gata5-Cre^* mutants in all cardiomyocytes, irrespective of Cre activation (Supplemental Figure 4, A–D). In control hearts at E10.5, sarcomeres, identified by cTnI antibody staining, appeared to be close to the cell membrane, as previously reported (28), in all cardiomyocytes (Figure 5, B and H). Fluorescence intensity analysis using ImageJ confirmed that in control embryos, cTnI staining was restricted close to the cardiomyocyte cell membrane, as shown by the two separate peaks at either side of the fluorescence intensity plot (Figure 5E). In contrast, in Cre-activated (GFP^+^) cardiomyocytes in *ROCKDN^Gata5-Cre^* mutants, the staining patterns of the sarcomeres were no longer restricted to the edges of the cells (Figure 5D); cTnI expression now appeared throughout the cell (Figure 5F). In contrast, staining patterns in Cre^–^ (GFP^–^) cardiomyocytes in the *ROCKDN^Gata5-Cre^* mutants were identical to the cardiomyocytes in control embryos, thus confirming that mislocalization of sarcomeric proteins at E10.5 was restricted to the cardiomyocytes in which ROCK function had been disrupted (Figure 5, G–J). To verify these data, we repeated the analysis using *ROCKDN^TnT-Cre^* mutants at E9.5 and E10.5, in which Cre was active throughout all of the cardiomyocytes. Staining at E9.5 showed comparable cTnI expression in the ventricular walls of control and *ROCKDN^TnT-Cre^* mutant embryos (Supplemental Figure 4, E–H). However, similar to the *ROCKDN^Gata5-Cre^* Cre-activated cardiomyocytes, in *ROCKDN^TnT-Cre^* mutants at E10.5, cTnI expression was mislocalized in all cardiomyocytes throughout the ventricular wall (Supplemental Figure 4, I–L). Therefore, we showed that loss of ROCK function by both mosaic cardiomyocyte expression of *Gata5-Cre* and uniform cardiomyocyte expression of *TnT-Cre* affected the intracellular structure of sarcomeres in embryonic cardiomyocytes at E10.5.

The article "Disruption of embryonic ROCK signaling reproduces the sarcomeric phenotype of hypertrophic cardiomyopathy" was retracted in 2020. Reason: fabricated or falsified data.

In order to confirm that the mislocalization of sarcomeres, first seen at E10.5, represented sarcomere disarray in *ROCKDN^Gata5-Cre^* cardiomyocytes, we examined sarcomeres at E10.5 by transmission electron microscopy (TEM). In control cardiomyocytes of the compact myocardium, the myofibrils were clearly defined, with long, continuous arrays of sarcomeric repeating units, separated by Z lines, and were generally found close to the cell membrane (Figure 5K). In comparison, sarcomeres in the *ROCKDN^Gata5-Cre^* mutants were dispersed throughout the cell and were disorganized (Figure 5L). The sarcomeric structures were quantified (29), and in *ROCKDN^Gata5-Cre^* mutants they were significantly longer and thinner than in control sarcomeres (Figure 5S), with significantly fewer repeating sarcomeric units per sarcomere (Figure 5T); the sarcomeres were separated by less-well-defined, diffuse Z lines (arrows in Figure 5N), which were significantly wider compared with control hearts (Figure 5U). In addition, there was structural myofibril discontinuity at the intercalated discs, which serve as the site of myofibril connection between neighboring cardiomyocytes, in the *ROCKDN^Gata5-Cre^* mutants. These myofibrils approached the intercalated disc at different angles, causing a disorganized or detached morphology (Figure 5, P and V). Within a single cardiomyocyte in the *ROCKDN^Gata5-Cre^* mutants, there was a mixture of normal and abnormal sarcomeres (Supplemental Figure 4, M and N). The destabilized structure of sarcomeres in the *ROCKDN^Gata5-Cre^* mutants suggests that the process of myofibrillogenesis may have been impaired, and was also associated with a reduction in myofibril density (Figure 5W) (30) and a significant increase in areas of G-actin accumulation (29) (which normally forms the F-actin of the thin filament; Figure 5, R and X). At E15.5, myofibrils in the *ROCKDN^Gata5-Cre^* mutants were again thinner and disjointed compared with the uniformly arranged sarcomeres in the control (Supplemental Figure 4, O and P). Likewise, in *ROCKDN^TnT-Cre^* mutants, TEM showed that the sarcomeres were abnormal at E10.5 (Supplemental Figure 4, Q and R). Taken together with the immunofluorescence data, this confirmed that downregulation of ROCK in cardiomyocytes caused disruption of sarcomere integrity in the ventricular wall as early as E10.5.

The article "Disruption of embryonic ROCK signaling reproduces the sarcomeric phenotype of hypertrophic cardiomyopathy" was retracted in 2020. Reason: fabricated or falsified data.

In order to establish whether disruption of sarcomeres by loss of ROCK signaling can trigger cardiomyocyte hypertrophy in a cell-autonomous manner, we used an in vitro approach. We cultured primary embryonic cardiomyocytes from control E17.5 embryos in serum-supplemented media and treated them with the ROCK inhibitor Y27632 (31). There was loss of sarcomeres, and the cardiomyocytes were significantly larger in ROCK inhibitor–treated cardiomyocytes compared with untreated control cardiomyocytes (Figure 6, A–C). Furthermore, the composition of the actin cytoskeleton was altered in the ROCK inhibitor–treated cardiomyocytes. There was a significant reduction in F-actin (stained by phalloidin; Figure 6, H and M) and an increase and altered cellular localization of G-actin (stained by DNase I; Figure 6, I–L). Therefore, this supports the idea that in vivo, reduced ROCK signaling altered the intracellular actin of the thin filaments and led to the early disruption of sarcomere structures, which may have subsequently led to the compensatory cardiomyocyte hypertrophy we observed at E16.5 onward in *ROCKDN^Gata5-Cre^* mutants.

### Disruption of sarcomere structure may be due to altered phosphorylation of the troponin complex.

As ROCK is known to phosphorylate the sarcomeric proteins cTnI, cTnT, and Mlc2 (3, 4) and because disruption of ROCK signaling in embryonic cardiomyocytes led to abnormal sarcomeric structure, we reasoned this may be linked to altered phosphorylation of these sarcomeric proteins. Therefore, we assessed whether phosphorylation of cTnI, cTnT, and Mlc2 was altered in the hearts of E13.5 *ROCKDN^Gata5-Cre^* mutants, using Pro-Q Diamond (Invitrogen) phosphoprotein stain, by determining the relative amount of phosphorylated protein to overall total protein concentration (Figure 7, A and B). As there are multiple bands on the Pro-Q gel, the same gel was transferred and blotted with the corresponding unphosphorylated antibodies to identify the correct band for analysis for each protein of interest (Figure 7C). *ROCKDN^Gata5-Cre^* hearts showed a significant decrease in the level of phosphorylated cTnI (ph-cTnI) and phosphorylated slow skeletal TnI (ph-ssTnI) expression (Figure 7, D and E) but no significant difference in ph-cTnT (Figure 7F). *ROCKDN^TnT-Cre^* mutants displayed a significant decrease in ph-cTnI, ph-ssTnI, and ph-cTnT (Figure 7, H–J). No change in phosphorylation of Mlc2 was observed in either *ROCKDN* mutant mouse line (Figure 7, G and K). These results were confirmed in vitro using protein extracted from primary mouse cardiomyocytes treated with the ROCK inhibitor Y27632. There was significantly reduced phosphorylation of cTnI, ssTnI, and cTnT, but not Mlc2 (Figure 7, L–O). Immunofluorescence using a phospho-specific TnI antibody confirmed reduced levels of ph-cTnI in Cre-activated cardiomyocytes at E10.5, prior to onset of a phenotype, in *ROCKDN^Gata5-Cre^* hearts (Figure 8, A–F). Thus, in the presence of ROCKDN protein, there was reduced phosphorylation of both isoforms of TnI and cTnT in embryonic cardiomyocytes.

co-IP confirmed that in embryonic hearts, ROCK1 and ROCK2 proteins bind to TnT, cTnI, and ssTnI (Figure 8, G and H), and that the interaction between ROCK1 and the 2 isoforms of TnI was significantly reduced in *ROCKDN^Gata5-Cre^* hearts (Figure 8, H–L). Thus, this may account for the reduced levels of phosphorylation observed in *ROCKDN^Cre^* hearts.

The article "Disruption of embryonic ROCK signaling reproduces the sarcomeric phenotype of hypertrophic cardiomyopathy" was retracted in 2020. Reason: fabricated or falsified data.

It is not clear whether phosphorylation of the troponin proteins is key to the formation of sarcomeres. To start to address this question, we treated control and *ROCKDN^Gata5-Cre^* primary cardiomyocytes with the drug IBMX, which is known to increase phosphorylation of TnI through the activation of protein kinase A (32). In control and *ROCKDN^Gata5-Cre^* Cre^–^ cardiomyocytes, IBMX did not significantly alter the average number of sarcomeres per cardiomyocyte (Figure 8, K, N, W, and Y). However, addition of IBMX significantly rescued the number of sarcomeres in *ROCKDN^Gata5-Cre^* Cre-activated cardiomyocytes from zero (Figure 8Q) to an average number of sarcomeres similar to that in control cardiomyocytes (Figure 8, T and Y). This suggests that the phosphorylation of the troponins may impact on sarcomere formation in embryonic cardiomyocytes.

### ROCKDN^Gata5-Cre^ mutant mice develop LV hypertrophy and dysfunction in adulthood.

Despite the presence of sarcomeric disruption and embryonic ventricular wall abnormalities, the *ROCKDN^Gata5-Cre^* mutant mice all survived to adulthood. Having established that cardiomyocytes in the *ROCKDN^Gata5-Cre^* mutant hearts were significantly hypertrophic compared with control hearts in late fetal development and postnatally (Figure 3), we extended this analysis to older mice to determine whether the hypertrophy persisted and if it increased further with age. At 4–12 months, cardiomyocytes in the *ROCKDN^Gata5-Cre^* mutant hearts continued to be significantly larger than those in control hearts at each time point (Figure 9, A and B, and Supplemental Table 3A). Interestingly, up to 4 months, the percent increase in cell size compared with control cardiomyocytes was similar in each of the 2 ventricles, but this became asymmetrical from 9 months. The increase in cardiomyocyte size in the LV increased significantly from 27% at 4 months to 43% at 9 months compared with only a nonsignificant increase from 22% to 30% in the RV. At 12 months, there was a further increase to 52% in the LV, while the RV remained at 31% (Figure 9, C and D, and Supplemental Table 3B). No corresponding increase in hypertrophy was seen in control hearts. Thus, there was a specific asymmetric increase in LV hypertrophy from 9 months.

The article "Disruption of embryonic ROCK signaling reproduces the sarcomeric phenotype of hypertrophic cardiomyopathy" was retracted in 2020. Reason: fabricated or falsified data.

Re-expression of fetal genes is associated with hypertrophy in cardiomyopathy (33), and therefore, we looked at gene expression levels in adult *ROCKDN^Gata5-Cre^* hearts from 1 to 12 months. A panel of genes were chosen that included fetal genes known to be re-expressed in ventricular hypertrophy (*ANF* and *Myh7*) and genes known to be dysregulated during hypertrophy (skeletal actin and phospholamban). In *ROCKDN^Gata5-Cre^* mutants, there was a significant increase in expression of *ANF* and *Myh7* and a significant decrease in expression of skeletal actin and phospholamban (Figure 9, E–H). These changes are all associated with hypertrophy and cardiac pathogenesis and coincide with the significant rise in hypertrophy observed at 9 months.

Antibody staining showed that sarcomeres were disrupted at E10.5 in *ROCKDN^Gata5-Cre^* mutant embryonic hearts, and therefore, we focused on the older hearts to establish whether this intracellular abnormality was retained. Clear sarcomeric staining was observed in control hearts (Figure 9I and Supplemental Figure 5, A–C), whereas there was loss of this staining throughout the heart in the *ROCKDN^Gata5-Cre^* mutants from P21 to 12 months (Figure 9J and Supplemental Figure 5, D–F). TEM analysis of 16-month hearts confirmed that there was disruption of the uniform pattern of repeating sarcomeres in *ROCKDN^Gata5-Cre^* mutant hearts (Supplemental Figure 5, G–J), and mutant sarcomeres were now significantly shorter and wider than in controls (Supplemental Figure 5, K and L).

The article "Disruption of embryonic ROCK signaling reproduces the sarcomeric phenotype of hypertrophic cardiomyopathy" was retracted in 2020. Reason: fabricated or falsified data.

Histological analysis of the adult hearts revealed there was no significant increase in fibrosis present until 9 months, at which point patches of interstitial fibrotic staining were seen in both the LV and RV, only in *ROCKDN^Gata5-Cre^* mutants, compared with control hearts (Figure 9, K–M, and Supplemental Figure 5, M–R). At each age there was positive staining in the valve tissue (data not shown). There was no accumulation of fat deposits in adult hearts (from 4 to 12 months) of *ROCKDN^Gata5-Cre^* mutants or controls (Supplemental Figure 5, S–V, and data not shown).

Despite the continued presence of intracellular abnormalities, increasing cellular hypertrophy, and fibrosis with age, *ROCKDN^Gata5-Cre^* mice appeared phenotypically healthy and indistinguishable from littermate controls at all ages. In order to assess whether these early cardiac developmental defects had any underlying impact on the adult heart, functional analysis was carried out by MRI. Reduced cardiac function was seen from 10 months in *ROCKDN^Gata5-Cre^* mutants, with a significant decrease in left (31.2 μl) and right (32.4 μl) stroke volumes (Figure 10, A and B); this resulted in significantly reduced cardiac output (Figure 10C), which also contributed to a reduction in heart rate at 16 months (Supplemental Figure 6A). End-diastolic LV wall thickness of *ROCKDN^Gata5-Cre^* mutants was significantly greater (Figure 10, D–F), with a corresponding decrease in end diastolic chamber diameter (Figure 10G), both from 10 months. Delta change in systolic-diastolic LV wall thickening was also significantly reduced (Figure 10H), and there was an overall significant increase in LV mass (Figure 10I), all from 10 months. No change in ejection fraction was observed (Supplemental Figure 6B). Analysis of the MRI images between 4 and 8 months showed that 67% of *ROCKDN^Gata5-Cre^* mutants had myocardial crypts in the LV wall, compared with 0% in the control mice (Supplemental Figure 6, C–F). These data demonstrate that the *ROCKDN^Gata5-Cre^* mutants developed LV concentric hypertrophy with systolic dysfunction as a consequence of the preexisting cellular hypertrophy and sarcomeric disruption.

## Discussion

We have shown that the early downregulation of ROCK signaling in a proportion of embryonic cardiomyocytes at E9.25 caused the disruption of sarcomeric structures in Cre-activated cardiomyocytes at E10.5. This led to reduced cardiomyocyte proliferation at E11.5 in *ROCKDN^Gata5-Cre^* hearts. In these mutant embryos, by E15.5, the compact wall of the ventricles was significantly thinner. Although, there was a significant increase in the thickness of the compact wall at E16.5, the ventricular wall of postnatal mutant hearts remained thinner, with increased presence of myocardial crypts. We propose that these intracellular abnormalities in sarcomeres, reduced cardiomyocyte proliferation, and delayed cardiomyocyte maturation led to the initiation of compensatory cardiomyocyte hypertrophy throughout the ventricular wall in late fetal stages of development, causing the abnormal ventricular myocardial wall development. The sarcomere disarray and cardiomyocyte hypertrophy persisted through postnatal and adult stages, causing re-expression of fetal genes, cardiac fibrosis, and concentric LV hypertrophic growth at 9 months, which ultimately impaired cardiac function from 10 months (Figure 11). Therefore, early disruption of embryonic sarcomeres led to cellular abnormalities and alterations in cardiac function, hence reproducing many of the clinical and histological features associated with the sarcomeric phenotype of HCM in patients.

The article "Disruption of embryonic ROCK signaling reproduces the sarcomeric phenotype of hypertrophic cardiomyopathy" was retracted in 2020. Reason: fabricated or falsified data.

Thus, the data presented here from our detailed analysis of *ROCKDN^Gata5-Cre^* mice provides convincing evidence for a novel developmental origin for HCM. Few studies have focused on establishing whether there are any embryonic defects in mouse models of HCM, and therefore the intracellular abnormalities in sarcomeric structure that we report here could have been missed. Mutations in *MYBPC3* account for a high proportion of HCM cases (33), and in the *Mybp3* KO mouse model, an embryonic phenotype was shown to predispose to HCM in adult mice (34). The study by Captur et al. focused on the emergence of structural abnormalities (the presence of myocardial crypts and abnormal trabecula patterns) in the ventricular wall during embryogenesis in their mutant mice, which were similar to our *ROCKDN^Gata5-Cre^* mutant embryos. However, they, did not examine the ultrastructure of embryonic sarcomeres or study the posttranslational modification of troponin proteins in cardiomyocytes, which we propose is the underlying embryonic trigger for the progression toward HCM in adulthood.

Mutations in the sarcomeric genes associated with HCM, including cardiac actin and troponins, are thought to disrupt the normal biophysical properties of the sarcomere, including sarcomere assembly (6). In *ROCKDN^Gata5-Cre^* mutants expression of ROCKDN led to the destabilization of the sarcomeres at E10.5. ROCK is well known to play a major role in regulating the rearrangement of actomyosin cytoskeleton (5) and myofibrillogenesis in cardiomyocytes, including the polymerization of G-actin into actin filaments (F-actin) (35). We showed that this process was impeded by reduced ROCK activity, shown by the increase in G-actin accumulation and abnormal sarcomeric structure in vivo and in vitro.

The article "Disruption of embryonic ROCK signaling reproduces the sarcomeric phenotype of hypertrophic cardiomyopathy" was retracted in 2020. Reason: fabricated or falsified data.

Structurally, both TnT and TnI are known to be required for the correct assembly of sarcomeres in early development (36–39), although it is not currently known whether phosphorylation of the troponins specifically influences sarcomere assembly in embryonic cardiomyocytes. There are 2 isoforms of TnI expressed in the heart, ssTnI and cTnI. ssTnI is the predominant embryonic and fetal isoform and is completely replaced by cTnI by 2–3 weeks postnatally (40). Interestingly, cTnI is first expressed at E10.5, which coincides which the emergence of the sarcomeric disruption observed in the *ROCKDN^Gata5-Cre^* embryos at this age. ROCK phosphorylates cTnI (S23, S24, and T144 in mouse and T143 in human *TNNI3*) and cTnT (S278 and T287 in mouse and S285 and T294 in human *TNNT2*), which impacts the function of myofilaments (4), and ROCK is predicted to phosphorylate ssTnI from in silico analysis (T51, S28, and S119) (41). Human HCM disease-causing mutations in residues R21 (R21C) and R145 (R145G and R145Q) in *TNNI3* were shown to specifically prevent the phosphorylation of these key residues (42). A mouse model of the R21C mutation linked reduced phosphorylation of cTnI to activation of the fetal gene program, hypertrophy and fibrosis in adult mice (43), which is similar to our findings in *ROCKDN^Gata5-Cre^* mice. The authors of the aforementioned studies, however, did not look at sarcomeric structure in their cells or embryonic hearts. By co-IP we confirmed that ROCK proteins bind to cTnT, cTnI, and ssTnI and this interaction was reduced in the presence of the ROCKDN protein, leading to reduced phosphorylation of these proteins in embryonic hearts. Preliminary studies shown here, using the drug IBMX (known to elevate intracellular cAMP levels, leading to an increase in phosphorylation of TnI; ref. 32) on primary *ROCKDN^Gata5-Cre^* cardiomyocytes, revealed a rescue of the structural integrity of sarcomeres in Cre-activated cardiomyocytes compared with untreated *ROCKDN^Gata5-Cre^* cardiomyocytes. Thus, this suggests for the first time to our knowledge that the phosphorylation of troponins by ROCK may be involved in sarcomere assembly in embryonic cardiomyocytes. It is hoped that future in vitro studies will establish how loss of phosphorylation by ROCK could directly lead to sarcomere disruption.

Similar to published mouse models of HCM (44) and disease progression in humans (45), the appearance of cardiac dysfunction and progression toward heart failure in our *ROCKDN^Gata5-Cre^* mice were delayed until adulthood. During development, there is normally a fetal phase of physiological hypertrophy, which along with cell proliferation, accounts for the heart growth seen before birth (28). We showed that in *ROCKDN^Gata5-Cre^* mutant embryos, there was a significant increase in hypertrophy in all cardiomyocytes, throughout the heart, from E16.5, which coincided with the increase in ventricular wall thickness at that age. We therefore hypothesize that in *ROCKDN^Gata5-Cre^* mutants, there was an excessive increase in this fetal phase of physiological hypertrophy compared with control embryos. This enabled the mutant hearts to compensate for the earlier delay in ventricular wall development, hence allowing the *ROCKDN^Gata5-Cre^* embryos to survive. Postnatally, the hypertrophic cardiomyocytes, throughout the whole heart from *ROCKDN^Gata5-Cre^* mutants, remained at approximately the same significantly increased level of physiological hypertrophy, with no impact on cardiac function up to 8 months. However, as the mouse matured further, this sustained persistent activation of compensatory hypertrophic responses eventually triggered pathological hypertrophy, which is known to be associated with maladaptive cardiac remodeling and gradual cardiac dysfunction (46). In HCM, this remodeling is specifically linked with an increase in LV hypertrophy, the upregulation of fetal gene expression, and the presence of interstitial fibrosis (all of which we saw at 9 months). This then leads to relaxation abnormalities in the heart (47) and an increase in LV mass and systolic dysfunction (which we saw at 10 months) in *ROCKDN^Gata5-Cre^* mutants. Furthermore, an increase in myocardial crypts was found in presymptomatic *ROCKDN^Gata5-Cre^* mice from E15.5 through to adulthood. This mirrors patients who are preclinical HCM mutation carriers, in whom cardiac structural abnormalities, including ventricular crypts (48) and abnormal trabecula patterning (49), have been identified.

The article "Disruption of embryonic ROCK signaling reproduces the sarcomeric phenotype of hypertrophic cardiomyopathy" was retracted in 2020. Reason: fabricated or falsified data.

Unexpectedly, we found that the expression level of the *ROCKDN* construct in the heart was significantly reduced to minimal levels from 3 months; hence ROCK function was only downregulated during embryogenesis and postnatally, and not in adulthood. This decrease in transcription is most likely due to the well-known epigenetic silencing of the CMV promoter by DNA methylation over time, as previously reported in mouse tissues (50–53). This is consistent with a previous report using the same *ROCKDN* transgenic mice, where there was no significant change in ROCK activity in 20-week-old hearts (19), suggesting that the expression of the *ROCKDN* construct had been silenced. Moreover, none of the previous publications using the *ROCKDN* mice have undertaken a detailed analysis of *ROCKDN* expression, as presented here, and therefore this phenomenon may have been missed. Furthermore, the expression level of endogenous *ROCK1* and *ROCK2* genes was not altered in *ROCKDN^Gata5-Cre^* mutants compared with controls. This was expected, as the ROCKDN protein forms homodimers with endogenous ROCK1 and ROCK2 proteins (54) and therefore does not impede the expression of the *ROCK* genes. In adult animal models where hypertrophy has been induced, the application of ROCK inhibitors has been associated with decreasing hypertrophy (55), suggesting a role for ROCK in regulating hypertrophy and in the transition from cardiac hypertrophy to heart failure (13, 56). However, this scenario is different from our *ROCKDN^Gata5-Cre^* model, as ROCK function was no longer downregulated in adult mice, and early embryonic disruption of ROCK was the developmental origin of the adult cardiomyopathy.

In one study, ROCK was linked to the development of a different form of cardiomyopathy, arrhythmogenic RV cardiomyopathy (ARVC) (19). The authors utilized the same *ROCKDN* transgenic mice used in our study, but under the control of either the *αMHC-Cre* (gave no phenotype) or the *SM22a-Cre* promoter, which gave rise to a model of ARVC. The progression to disease differed from that in our *ROCKDN^Gata5-Cre^* mice, as they had a severe postnatal phenotype and features associated with ARVC. In comparison to their results, we did not find any myocardial fibrofatty changes; no increase in expression of *Cnntb1*, *Wnt5b*, or *PPARγ*; and no desmosomal abnormalities (Supplemental Figure 7). The discrepancy between the 2 models is most likely due to the influence of different genetic backgrounds (57) and the different expression patterns of the Cre promoters. *SM22α* is expressed in the heart tube from E8.0, but expression decreases in the heart from E10.5, with no cardiac expression by E13.5, and becomes restricted to the smooth muscle cells of the vasculature and visceral organs (58). In the *Gata5-Cre* and *Tnt-Cre* lines used in our study, *Cre*, and hence *ROCKDN*, is expressed in cardiomyocytes throughout development. Therefore, the sarcomere disarray we observed at E10.5 persisted throughout development, spreading to the whole heart, which would more likely mimic the consequences of a sarcomeric mutation in a patient who develops HCM.

As the clinical presentation of HCM is very heterogeneous, it is even more important that the underlying complex pathophysiology of this disease is understood. Our study highlights that there is a developmental origin for HCM and the possibility that undetected nonlethal embryonic ventricular wall defects can predispose to cardiomyopathy later in life. Hence, it is important to unravel how early intracellular defects in the embryonic cardiomyocytes can go undetected and manifest as cardiovascular disease. Thus, the identification of additional genetic variants in presymptomatic patients will provide individualized prognostic information and ensure early clinical investigations, which may show early signs of structural or functional abnormalities, allowing targeted treatment to be developed. The *ROCK* genes are therefore potential candidate genes to add to the panel of genes screened routinely in HCM patients.

The article "Disruption of embryonic ROCK signaling reproduces the sarcomeric phenotype of hypertrophic cardiomyopathy" was retracted in 2020. Reason: fabricated or falsified data.

## Methods

Further information can be found in Supplemental Methods, available online with this article.

### Mice.

Transgenic ROCK dominant-negative (*ROCKDN*) mice (15) were intercrossed with the *R26ReYFP* reporter line (25). Cardiac-specific *Cre* lines were used to target ROCK downregulation in the myocardium using *TnT-Cre* (22), the myocardium and epicardium using *Gata5-Cre* (23), and the epicardium using *WT1-ERT-Cre* (24). Genotyping primers are shown in Supplemental Table 1.

*H&E, Sirius red, and oil red O staining*. H&E and Sirius red staining were performed following standard protocols. Sirius red fluorescence was detected using the rhodamine channel (excitation 538–562 nm, emission 570–640 nm) (59), allowing quantification of fibrosis within a tissue by measuring fluorescence intensity using ImageJ (NIH) software. A total of 3 tissue-matched sections were analyzed per sample. Oil red O staining was performed to assess lipid content within heart sections following standard protocols. Slides were imaged using an Axio Imager 2 (Zeiss).

### Immunofluorescence and immunohistochemistry.

Staining was performed on paraffin-fixed embryonic and postnatal hearts, and cryosections from adult hearts. Sections were incubated with primary antibody overnight at 4°C. Sections were washed and incubated with the appropriate secondary antibody. Slides were imaged using Axio Imager 2 and a Nikon A1R confocal. Antibodies are detailed in Supplemental Table 2.

### Cardiomyocyte proliferation.

Cardiomyocyte proliferation was analyzed in embryonic hearts by BrdU incorporation. Pregnant dams were given an i.p. injection of 25 mg/ml BrdU (MilliporeSigma) 1 hour prior to sacrifice. Embryos were fixed in paraformaldehyde at 4°C overnight, then processed through an ethanol series and embedded in paraffin. 8-μm tissue sections were collected, and IF was performed using BrdU antibody: Cre-activated cells were stained with GFP antibody and counterstained with DAPI. Cell counts were performed on 3 matched tissue sections for each sample. Between 2000 and 2500 cells were counted in both the LV and RV for each embryo, and the average was calculated.

The article "Disruption of embryonic ROCK signaling reproduces the sarcomeric phenotype of hypertrophic cardiomyopathy" was retracted in 2020. Reason: fabricated or falsified data.

### qRT-PCR.

Total RNA was isolated using the ReliaPrep RNA Miniprep System (Promega, catalog Z6010). cDNA was synthesized using a High-Capacity cDNA reverse transcription kit (Applied Biosystems, catalog 4368814). qRT-PCR was performed using fast SYBR green mastermix (Life Technologies). Relative quantities of gene expression were calculated and were normalized to the housekeeping gene *Gapdh*. qRT-PCR primers are listed in Supplemental Table 3.

### Cardiomyocyte isolation.

Primary cardiomyocytes were isolated from embryonic E15.5 or E17.5 hearts and treated with the ROCK inhibitor Y27632 or IBMX, as detailed in the Supplemental Methods.

### TEM.

TEM was performed on E10.5 and E15.5 embryonic and 16-month adult heart tissue (Philips CM100; Electron Microscopy Research Services, Newcastle University) to assess sarcomere structure.

### High-resolution episcopic microscopy.

E15.5 embryos were collected and processed, and high-resolution episcopic microscopy (HREM) imaging was performed in-house (60).

### Phosphoproteomics.

Total protein was prepared from E13.5 embryonic hearts (individual younger hearts did not provide sufficient protein required for this assay), and primary cardiomyocytes, in 100 μl CelLytic buffer (MilliporeSigma, C2978) with protease and phosphatase inhibitors. Western blot analysis was performed. Protein (20 μg) was separated via SDS-PAGE, transferred to a nitrocellulose membrane, and probed with primary antibodies (Supplemental Table 4). Membranes were incubated with the secondary antibody and visualized via ECL using the LI-COR C-DiGit. Phosphorylated protein was assessed using Pro-Q Diamond in-gel staining assay (Invitrogen, P33300) following the manufacturer’s instructions (61). Once stained, the gels were imaged, and the amount of phosphorylated protein present was calculated. The gel was then stained with Coomassie blue (MilliporeSigma, B0770), allowing total protein to be calculated. The amount of phosphorylated protein relative to total protein was calculated using ImageJ.

### IP.

Co-IP was performed with primary antibody immobilized onto magnetic Dynabeads Protein G or A (Invitrogen, 10007D) and incubated with total protein lysates from E16.5 control and *ROCKDN^Gata5-Cre^* hearts overnight at 4°C. Supernatants were discarded, beads were washed and then protein was eluted and collected. Western blot analysis was then performed. Samples were then run on 4-12% Bis-Tris protein gels (Invitrogen, NP0322BOX) and probed using the appropriate antibody (Supplemental Table 4).

### MRI.

Cardiac cine MRI was performed as previously described (62). Scans were then converted to matfiles using MATLAB script and LV and RV function analyzed using the freely available software Segment v1.8 (http://segment.heiberg.se).

The article "Disruption of embryonic ROCK signaling reproduces the sarcomeric phenotype of hypertrophic cardiomyopathy" was retracted in 2020. Reason: fabricated or falsified data.

### ECG.

Heart rate was measured in adult mice using a 3-lead ECG as described previously (63), and analysis was performed using LabChart software (ADInstruments).

### Statistics.

A normality test (Shapiro-Wilk) was performed on all the data. For nonparametric data, a Mann-Whitney *U* test was used, and for parametric data either an unpaired *t* test or 1-way ANOVA with Bonferroni’s correction for multiple comparisons was performed. A χ^2^ test was used to analyze Mendelian numbers. In all graphs, data are presented as mean ± SEM. Significance was deemed as *P* < 0.05. Analyses were performed using GraphPad Prism software (version 7.01).

### Study approval.

All mouse experiments were performed in accordance with the Animals (Scientific Procedures) Act 1986, United Kingdom, under project license PPL PC7996264. All experiments were approved by the Newcastle University Ethical Review Panel.

## Author contributions

HMP designed the research study, analyzed the data, and wrote the manuscript. KEB conducted the majority of the experiments, acquired the data and images, and wrote the methods. GAM analyzed the MRI data and wrote that part of the manuscript. STC helped perform the MRI studies and analyze the data. LP helped perform experiments, and TJM carried out the HREM experiments and generated the images. HMA, DJH, and SDB were involved in discussions and analysis of data throughout the duration of the project, and helped review and edit the manuscript.

## Supplementary Material

Supplemental data

## Figures and Tables

**Figure 1:** Downregulation of ROCK1 and ROCK2 in embryonic cardiomyocytes leads to defects in the ventricular wall during embryogenesis. (**A**–**L**) Transverse sections from embryos were stained with H&E, and a representative high-power image of the right ventricle is shown for each genotype and embryonic age. At E10.5, the heart morphology was comparable among controls (**A**) and *ROCKDN^TnT-Cre^* (**E**) and *ROCKDN^Gata5-Cre^* (**I**) mutants. A reduction in myocardial thickness was visually evident throughout both ventricles at E11.5 in *ROCKDN^TnT-Cre^* (arrow in **F**) and *ROCKDN^Gata5-Cre^* (arrow in **J**) mutant hearts compared with control hearts (**B**). Reduced myocardial thickness was still present at E15.5 in *ROCKDN^TnT-Cre^* (**G** and **H**) and *ROCKDN^Gata5-Cre^* (**K** and **L**) mutants compared with control hearts (**C** and **D**). The *ROCKDN^TnT-Cre^* mutants had no defined interventricular sulcus (arrow in **G**). The severity of myocardial wall thickness was more prominent in *ROCKDN^TnT-Cre^* hearts than *ROCKDN^Gata5-Cre^* mutants (compare arrows in **H** and **L**). (**M** and **N**) Myocardial wall measurements confirmed that the compact myocardium was significantly thinner in *ROCKDN^TnT-Cre^* mutants at E12.5*,* E14.5, and E15.5 (**M**), and at E14.5 and E15.5 in *ROCKDN^Gata5-Cre^* mutants (**N**), compared with littermate control embryos. E10.5 *n* = 5, E11.5 *n* = 5, E12.5 *n* = 5, E14.5 *n* = 5, E15.5 *n* = 5 for *ROCKDN^TnT-Cre^* mutants and littermate controls; and E10.5 *n* = 6, E11.5 *n* = 6, E12.5 *n* = 6, E14.5 *n* = 5, E15.5 *n* = 12 for *ROCKDN^Gata5-Cre^* mutants and littermate controls. Data are presented as mean ± SEM. **P < 0.01, ****P < 0.0001 by 1-way ANOVA with Bonferroni’s correction for multiple comparisons. rv, right ventricle; lv, left ventricle. Scale bars: 100 μm.

The article "Disruption of embryonic ROCK signaling reproduces the sarcomeric phenotype of hypertrophic cardiomyopathy" was retracted in 2020. Reason: fabricated or falsified data.

**Figure 2:** Impaired maturation of the ventricular wall in late fetal and postnatal *ROCKDN^Gata5-Cre^* mutants. (**A** and **B**) Measurements of the compact myocardial wall were performed on transverse heart sections from E15.5 (*n* = 12), E16.5 (*n* = 5), and E17.5 (*n* = 4) embryos, and P0 (*n* = 3), P4 (*n* = 3), P7 (*n* = 3), and P21 (*n* = 4) postnatal pups, in both the left ventricle (**A**) and right ventricle (**B**), in control and *ROCKDN^Gata5-Cre^* mutant littermates. During embryonic and postnatal development, generally, the compact myocardium of the control hearts is thicker than in mutant hearts. In particular, in the left ventricle, the control compact myocardium is significantly thicker than in the *ROCKDN^Gata5-Cre^* mutant compact myocardium at E15.5, P4, P7, and P21 (**A**); and in the right ventricle it is significantly thicker at E15.5, P7 and P21 (**B**). From E15.5 to E16.5 in *ROCKDN^Gata5-Cre^* mutant hearts, myocardial wall thickness increased significantly, in both the left ventricle and right ventricle (red lines), whereas no corresponding significant increase was observed in control hearts (blue lines). (**C**–**F**) High-resolution episcopic microscopy imaging at E15.5 showed that *ROCKDN^Gata5-Cre^* hearts (**D** and **F**) displayed an immature thin myocardial wall containing myocardial crypts within the compact myocardium (red arrows **F**) compared with controls (**C** and **E**). *n* = 10 for each genotype. (**G**–**J**) Phenotypic analysis of 4-chamber view sections from postnatal hearts, stained with the histological stain H&E, confirmed that in the *ROCKDN^Gata5-Cre^* hearts the ventricular wall was visibly thinner and that it also contained myocardial crypts (arrows) at P0 and P21. *n* = 3 for each genotype at each time point. (**K**) Trabecular complexity for each heart was assessed by calculating the ratio of trabecular myocardial area to compact myocardium area throughout the ventricles. There were no significant differences between control and mutant hearts during fetal and postnatal development, confirming that *ROCKDN^Gata5-Cre^* mutants did not have a non-compaction phenotype. E15.5 (*n* = 8), E17.5 (*n* = 6), P0, and P21 (*n* = 3) for each genotype at each time point. Data are presented as mean ± SEM. *P < 0.05, **P < 0.01, ***P < 0.001, ****P < 0.0001 by 1-way ANOVA with Bonferroni’s correction for multiple comparisons. lv/LV, left ventricle; rv/RV, right ventricle. Scale bars: 100 μm.

The article "Disruption of embryonic ROCK signaling reproduces the sarcomeric phenotype of hypertrophic cardiomyopathy" was retracted in 2020. Reason: fabricated or falsified data.

**Figure 3:** Reduced proliferation of cardiomyocytes followed by increased cardiomyocyte hypertrophy leads to abnormal ventricular wall development in *ROCKDN^Gata5-Cre^* mutants. (**A** and **B**) Transverse sections from control and *ROCKDN^Gata5-Cre^* mutant embryos collected from mothers injected with BrdU were stained with BrdU antibody to label proliferating cells (green staining) and GFP antibody to stain Cre-activated cells (red staining). The total number of Cre-activated cardiomyocytes and total number of proliferating Cre-activated cardiomyocytes, in which ROCK was downregulated, were determined in each sample, from which the percentage of proliferating Cre-activated cardiomyocytes was calculated. A representative image of the left ventricle from E11.5 embryos is shown. (**C**) No significant difference in the percentage of proliferating Cre-activated cardiomyocytes was detected in the left or right ventricle at E10.5. At E11.5 there was a significant decrease in the percentage of proliferating Cre-activated cardiomyocytes in *ROCKDN^Gata5-Cre^* mutants, in both the left and right ventricles compared with controls. *n* = 6 for each genotype at both time points. (**D**) No significant difference in cardiomyocyte proliferation was identified in *ROCKDN^Gata5-Cre^* hearts at either E15.5 or E16.5. *n* = 3 for each genotype at both time points. (**E**) The average number of cardiomyocytes in the compact myocardium, per field of view, was calculated at E15.5, E16.5, and E17.5 and showed a significant decrease in the number of cardiomyocytes in *ROCKDN^Gata5-Cre^* hearts at E16.5 and E17.5 in both the left and right ventricle, compared with controls. *n* = 3 for each genotype at all time points. (**F** and **G**) Wheat germ agglutinin (WGA) immunofluorescence was used to determine cardiomyocyte cell size in control and *ROCKDN^Gata5-Cre^* hearts. The cardiomyocytes in *ROCKDN^Gata5-Cre^* hearts (**G**) were visibly larger than those in control hearts (**F**). In *ROCKDN^Gata5-Cre^* hearts, both Cre-activated/GFP^+^ (GFP+ve) (green staining) (example cell outlined in yellow in **H**–**J**) and GFP^–^ (GFP-ve; example cell outlined in white cell in **H**–**J**) cardiomyocytes were hypertrophic. (**K** and **L**) In *ROCKDN^Gata5-Cre^* hearts, the cardiomyocytes in the compact myocardium were significantly larger compared with control hearts, from E16.5 to P21 in the left ventricle (**K**) and from E15.5 to P7 in the right ventricle (**L**). *n*=5 for E15.5 and E16.5; *n* = 4 for E17.5 and P21; *n* = 3 for P0, P4, and P7 for each genotype. Data are presented as mean ± SEM. *P < 0.05, **P < 0.01, ***P < 0.001, ****P < 0.0001 by 1-way ANOVA with Bonferroni’s correction for multiple comparisons. lv/LV, left ventricle; RV, right ventricle. Scale bars: 100 μm (**A** and **B**), 50 μm (**F** and **G**), and 20 μm (**H**–**J**).

The article "Disruption of embryonic ROCK signaling reproduces the sarcomeric phenotype of hypertrophic cardiomyopathy" was retracted in 2020. Reason: fabricated or falsified data.

**Figure 4:** Delayed maturation of cardiomyocytes in *ROCKDN^Gata5-Cre^* mutants. (**A**–**E**) The pattern of α-SMA expression was investigated by immunohistochemistry and visualized by DAB staining, and a representative image of the left ventricular wall, from each age, is shown. In control hearts at E15.5 and E17.5, α-SMA became restricted to the compact myocardium and was no longer expressed in trabeculae (arrows in **A** and **B**). Postnatally, expression was further restricted to the smooth muscle of coronary arteries, with no cardiomyocyte staining by P7 (**C**–**E**). In contrast, in *ROCKDN^Gata5-Cre^* mutants, α-SMA staining persisted in trabeculae at E15.5 and E17.5 (arrows in **F** and **G**), and there were patches of cardiomyocyte expression postnatally (arrows in **H**–**J**). (**K**) The level of α-SMA expression was measured by ImageJ in trabeculae and in the compact myocardium. The total area of trabeculae or the compact myocardium was measured throughout the heart, and the percentage of this area in which α-SMA was expressed was calculated. This confirmed that α-SMA expression was retained longer in trabeculae in *ROCKDN^Gata5-Cre^* mutants, as there were significantly higher levels of α-SMA expression at E15.5 and E17.5 in trabeculae of mutants compared with trabeculae of littermate controls. Furthermore, in control hearts at E15.5, there was a significant difference in α-SMA expression levels between trabeculae and the compact myocardium (blue line), confirming, as expected, that the expression was becoming restricted to the compact myocardium. In contrast, in *ROCKDN^Gata5-Cre^* mutants, there was no significant difference between expression levels in trabeculae and compact myocardium (purple line; NS). By E17.5, there was a significant difference in expression levels in the compact myocardium between controls and mutants, showing that, as expected, expression in control hearts was beginning to decrease in the compact myocardium as the cardiomyocytes matured and that this process was delayed in *ROCKDN^Gata5-Cre^* mutants. *n* = 8 for E15.5 and *n* = 6 for E17.5 for each genotype. Data are presented as mean ± SEM. *P < 0.05, **P < 0.01, ****P < 0.0001 by 1-way ANOVA with Bonferroni’s correction for multiple comparisons. lv, left ventricle. Scale bars: 100 μm.

The article "Disruption of embryonic ROCK signaling reproduces the sarcomeric phenotype of hypertrophic cardiomyopathy" was retracted in 2020. Reason: fabricated or falsified data.

**Figure 5:** Destabilization of sarcomeres in *ROCKDN^Gata5-Cre^* mutant cardiomyocytes at E10.5. (A–J) Transverse sections from E10.5 embryos were stained by immunofluorescence to identify all cardiomyocytes (cTnI staining, green) and Cre-activated cardiomyocytes/GFP^+^ cells (red staining). In Cre-activated cardiomyocytes of control embryos, cTnI was cortical (red arrows in **B**), confirmed by the 2 separate curves in the fluorescence intensity profile plot (**E**). In contrast, in Cre-activated cardiomyocytes of *ROCKDN^Gata5-Cre^* mutants, cTnI staining was disrupted, as it was diffuse throughout the cell (red arrows in **D**), confirmed by the continuous line in the fluorescence intensity profile plot (**F**). The cTnI staining in GFP negative cardiomyocytes in control and *ROCKDN^Gata5-Cre^* mutants was identical (white arrows in **G**–**J**). *n*=6 for each genotype. (**K**–**R**) Representative TEM imaging of myofibrils at E10.5. In controls, the sarcomeres generally align in close proximity to the plasma membrane and are highly organized (arrows in **K**). In *ROCKDN^Gata5-Cre^* cardiomyocytes, the myofibrils are located throughout the cells and show sarcomere collapse (arrows in **L**). The average width of the Z discs throughout the sarcomeres was significantly increased in *ROCKDN^Gata5-Cre^* cardiomyocytes compared with controls (**M**, **N**, and **U**). Myofibril discontinuity was present at cellular junctions in *ROCKDN^Gata5-Cre^* as the myofibrils approached the intercalated discs at more varied wider angles (arrows in **P** and **V**) but not seen in controls (**O**). Areas of G-actin accumulation were detected in *ROCKDN^Gata5-Cre^* cardiomyocytes (**R**) more frequently that in control hearts (**Q**) giving a significant increase in G-actin density (**X**). (**S**) There was a significant increase in sarcomere length and decrease in sarcomere width in *ROCKDN^Gata5-Cre^* mutants compared with sarcomeres in control hearts. (**T**) The number of repeating sarcomeric units, per field of view in comparative regions, was significantly reduced in *ROCKDN^Gata5-Cre^* cardiomyocytes. (**W**) As a consequence of the abnormal sarcomeric structure, in *ROCKDN^Gata5-Cre^* cardiomyocytes, there was significantly reduced myofibril density per field of view. (**X**) The percent area containing G-actin, per field of view, showed a significant increase in *ROCKDN^Gata5-Cre^* cardiomyocytes. *n* = 5 for each genotype. lv, left ventricle; pm, plasma membrane. Data are presented as mean ± SEM. **P < 0.01, ***P < 0.001, ****P < 0.0001 by unpaired *t* test. Scale bars: 50 μm (**A**–**D** and **G**–**J**) and 500 nm (**K**–**R**).

The article "Disruption of embryonic ROCK signaling reproduces the sarcomeric phenotype of hypertrophic cardiomyopathy" was retracted in 2020. Reason: fabricated or falsified data.

**Figure 6:** Loss of sarcomere structure and increased hypertrophy in primary cardiomyocytes after treatment with the ROCK inhibitor Y27632. Primary cardiomyocytes from E17.5 control embryos were cultured, and half were treated with the ROCK inhibitor Y27632. Cardiomyocytes were identified by staining with cTnI antibody, which stains sarcomeres (green). In the control group, the organized structure of the sarcomeres was clearly visible (**A**), whereas addition of Y27632 abolished the sarcomeric structure, and the cardiomyocytes appeared hypertrophic (**B**) compared with untreated control cardiomyocytes. (**C**) Cardiomyocyte area was calculated using ImageJ. The average cell area was calculated from a total of 10 cells from each treatment group, and the measurements confirmed that there is a significant increase in cell size with the addition of Y27632. *n*=4. (**D**–**I**) To analyze the actin composition of the cultured cardiomyocytes, we stained for G-actin (DNase I, green staining) and F-actin (phalloidin, red staining). Staining of both phalloidin (**H**) and DNase I (**I**) was disrupted in Y27632-treated cardiomyocytes, with loss of F-actin in the cytoplasm and an accumulation of DNase I around the nuclear membrane, illustrated by the fluorescence intensity profile plots (**J** and **K**). Fluorescence intensity measurements confirmed there was a significant increase in DNase I staining (**L**) and a decrease in phalloidin staining (**M**). *n* = 3 biological replicates for primary cardiomyocytes. Data are represented as mean ± SEM. *P < 0.05, **P < 0.01, ***P < 0.001 by unpaired *t* test. Scale bars: 20 μm (**A**, **B**, and **D**–**I**).

**Figure 7:** Downregulation of ROCK function leads to decreased phosphorylation of TnI and cTnT in vivo and in vitro. Pro-Q Diamond phosphoprotein stain was used to determine the total amount of the phosphorylated form of each protein (**A**), and Coomassie blue was used to determine total amount of each protein (**B**) at E13.5 in control, *ROCKDN^Gata5-Cre^*, and *ROCKDN^TnT-Cre^* mutant hearts and in isolated primary mouse cardiomyocytes treated with and without the ROCK inhibitor Y27632. Representative gel images are shown for each type of sample analyzed. (**C**) Western blot analysis of the same blot shown in **A** and **B**, using specific antibodies, confirmed that the correct bands on the Pro-Q and Coomassie blue blots (arrows in **A** and **B**) were measured by densitometry for the proteins of interest: cTnT 40 kDa, cTnI 26 kDa, ssTnI 22 kDa, and Mlc2 18 kDa. (**D**–**O**) The relative amount of phosphorylated protein to total protein was calculated using densitometry for control and mutant heart or cell samples. A significant reduction in ph-cTnI and ph-ssTnI was observed in *ROCKDN^Gata5-Cre^* (**D** and **E**) compared with controls. A significant reduction in ph-cTnI, ph-ssTnI, and additionally ph-TnT was observed in *ROCKDN^TnT-Cre^* mutants (**H**–**J**) compared with controls. Primary cardiomyocytes from E17.5 control embryos treated with Y27632 also showed a significant reduction in ph-cTnI (**L**), ph-ssTnI (**M**), and ph-TnT (**N**). No change in the levels of ph-Mlc2 was observed in any of the groups (**G**, **K**, and **O**). *n* = 4 for each genotype and *n* = 3 biological replicates for primary cardiomyocytes. Data are presented as mean ± SEM. *P < 0.05, **P < 0.01 by unpaired *t* test. CM, cardiomyocytes.

The article "Disruption of embryonic ROCK signaling reproduces the sarcomeric phenotype of hypertrophic cardiomyopathy" was retracted in 2020. Reason: fabricated or falsified data.

**Figure 8:** Reduction in binding between ROCK and TnI proteins may account for reduced ph-TnI expression in *ROCKDN^Gata5-Cre^* mutants, and increased phosphorylation by IBMX rescues the sarcomeric phenotype in vitro. (**A**–**C**) Immunofluorescence staining of ph-cTnI (green) in Cre-activated/GFP^+^ cells (red staining) in cardiomyocytes of control E10.5 hearts (yellow arrows). (**D**–**F**) There was a reduction in ph-cTnI staining in Cre-activated cardiomyocytes in *ROCKDN*^Gata5-Cre^ hearts (white arrows) compared with control samples (yellow arrows). *n* = 3 for each genotype. (**G** and **H**) Co-IP using protein extracts from whole heart lysates from E16.5 embryos showed that in control hearts, ROCK1 (158kDa) and ROCK2 (161 kDa), bind to cTnT (40 kDa) (**G**) and to cTnI (26 kDa) and ssTnI (22 kDa) (**H**). (**I**) In *ROCKDN^Gata5-Cre^* mutant hearts, there was a significant reduction in binding between the ROCK proteins and the troponin proteins. Co-IP with TnI showed a significant reduction in expression of ROCK1 and ROCK2, and conversely, in the same samples, co-IP with ROCK1 gave a significant reduction in cTnI and ssTnI expression in *ROCKDN^Gata5-Cre^* mutants. *n* = 4 for each genotype. (**J**–**X**) Primary cardiomyocytes were cultured from E15.5 control and *ROCKDN^Gata5-Cre^* mutants. GFP antibody was used to identify the Cre-activated (Cre+ve) cells (red staining), and cTnI antibody confirmed which cells were cardiomyocytes by labeling sarcomeres (green). Addition of IBMX to control cells did not have any effect (**M**–**O**). Cre-activated cardiomyocytes from *ROCKDN^Gata5-Cre^* mutants, lacked sarcomeric structure (**P**–**R**). Addition of IBMX rescued the sarcomeric structure in Cre-activated cardiomyocytes from *ROCKDN^Gata5-Cre^* mutants (**S**–**U**). Similar to the control samples, Cre^–^ cells from *ROCKDN^Gata5-Cre^* mutants had normal sarcomeric organization that was not altered following the addition of IBMX (**V**–**X**). (**Y**) The average number of sarcomeres per cardiomyocyte, from a total of 10 cells per well, was determined. There were no significant differences between control Cre^+^ cardiomyocytes with and without IBMX. There was a significant difference in sarcomere number between *ROCKDN*^Gata5-Cre^ Cre^+^ cardiomyocytes without IBMX compared with both control samples. Addition of IBMX to *ROCKDN*^Gata5-Cre^ Cre^+^ cardiomyocytes significantly increased sarcomeres, to a level that was no longer significantly different relative to both control groups; thus, addition of IBMX rescues the sarcomeric phenotype of *ROCKDN*^Gata5-Cre^ Cre^+^ cardiomyocytes. *n* = 3 for each genotype. Data are presented as mean ± SEM. *P < 0.05, **P < 0.01 by unpaired *t* test (**I**) and ****P < 0.0001 by 1-way ANOVA with Bonferroni’s correction for multiple comparisons (**Y**). Scale bars: 50 μm (**A**–**F**) and 10 μm (**J**–**X**).

The article "Disruption of embryonic ROCK signaling reproduces the sarcomeric phenotype of hypertrophic cardiomyopathy" was retracted in 2020. Reason: fabricated or falsified data.

**Figure 9:** Adult *ROCKDN^Gata5-Cre^* mutants develop left ventricular hypertrophy, fibrosis, and re-expression of fetal genes from 9 months. (**A** and **B**) Four-chamber-view sections of dissected hearts from P21 and 4-, 9-, and 12-month control and *ROCKDN^Gata5-Cre^* mutants were stained with WGA to allow the average area of the cardiomyocytes to be calculated from left (**A**) and right (**B**) ventricles. In the left ventricle, cardiomyocytes were significantly larger in *ROCKDN^Gata5-Cre^* mutants compared with controls at all ages, and in the right ventricle cardiomyocytes were significantly larger from 4 months (black lines). The average percent increase in cardiomyocyte size in *ROCKDN^Gata5-Cre^* mutants compared with controls was calculated. In the *ROCKDN^Gata5-Cre^* mutants, there was a significant change from 4 to 9 months (from 27% to 43%) and from 9 to 12 months (43% to 52%) in the left ventricle (**C**), with no corresponding significant increase in the right ventricle (**D**). Hence, there was a specific increase in left ventricular hypertrophy in the *ROCKDN^Gata5-Cre^* mutants. *n*=4 P21, *n* = 3 4 months, *n* = 5 9 and 12 months, for each genotype. (**E**–**H**) qRT-PCR was used to detect any significant changes in gene expression using cDNA isolated from dissected hearts. In *ROCKDN^Gata5-Cre^* mutants, compared with control hearts, there was a significant increase in the relative expression of fetal genes *ANF* and *Myh7* from 9 months; and a significant decrease in expression of skeletal actin and phospholamban, which are dysregulated during hypertrophy. (**I** and **J**) Immunofluorescence staining with cTnI (green) showed disruption in sarcomere striations at 9 months throughout the heart in *ROCKDN^Gata5-Cre^* mutants (**J**) compared with controls (**I**). (**K** and **L**) Patches of fibrosis were seen throughout the heart from 9 months, and there was a significant increase in the levels of fibrosis, calculated from fluorescence intensity measurements, in both ventricles at 9 and 12 months (**M**). *n* = 3 for each genotype at each time point for experiments in **E**–**M**. Data are presented as mean ± SEM. *P < 0.05, **P < 0.01, ***P < 0.001, ****P < 0.0001 by 1-way ANOVA with Bonferroni’s correction for multiple comparisons. lv/LV, left ventricle; RV, right ventricle; M, month. Scale bars: 50 μm (**I** and **J**) and 100 μm (**K** and **L**).

The article "Disruption of embryonic ROCK signaling reproduces the sarcomeric phenotype of hypertrophic cardiomyopathy" was retracted in 2020. Reason: fabricated or falsified data.

**Figure 10:** *ROCKDN^Gata5-Cre^* mutants have features of hypertrophic cardiomyopathy, with increased left ventricular mass and reduced cardiac function from 10 months. Heart function was assessed by cine cardiac MRI in mice aged 4–16 months. This identified a significant reduction in left (**A**) and right (**B**) ventricle stroke volume at 10 and 16 months in *ROCKDN^Gata5-Cre^* compared with control hearts, with an overall significant reduction in cardiac output also from 10 months in *ROCKDN^Gata5-Cre^* mutants compared with controls (**C**). (**D**–**F**) In MRI images, the left ventricular wall appears thicker in *ROCKDN^Gata5-Cre^* mutants compared with controls (white lines in **D** and **E**). Measurements confirmed that there was a significant increase in end-diastolic left ventricular wall thickness in *ROCKDN^Gata5-Cre^* hearts (**F**), with a corresponding significant decrease in end-diastolic chamber diameter (**G**), and a significant reduction in delta change in systolic-diastolic left ventricular wall thickness (**H**) compared with controls, all from 10 months. There was an overall significant increase in LV mass/body weight ratio from 10 months (**I**) compared with controls. *n* = 3 for 4 months, *n* = 3 for 6 months, *n* = 3 for 8 months, *n* = 5 for 10 months, *n* = 8 for 16 months, for each genotype. Data are presented as mean ± SEM. *P < 0.05, **P < 0.01, ****P < 0.0001 by 1-way ANOVA with Bonferroni’s correction for multiple comparisons. M, month.

**Figure 11:** Loss of ROCK function in embryonic cardiomyocytes causes sarcomere disarray, leading to defects in ventricular wall development and compensatory fetal hypertrophy, predisposing to left ventricular hypertrophy, and ultimately HCM in adulthood. Disruption of ROCK signaling in embryonic cardiomyocytes in *ROCKDN^Gata5-Cre^* mutants led to disruption of the sarcomeric structure and reduced phosphorylation of cTnI, ssTnI, and cTnT at E10.5. This reduced cell proliferation at E11.5 delayed cardiomyocyte maturation, resulting in compensatory fetal hypertrophy of the cardiomyocytes throughout the heart by E16.5. The ventricular wall was significantly thinner and contained myocardial crypts between trabeculae, which along with hypertrophy and disruption of sarcomeric structure continued throughout the life of the *ROCKDN^Gata5-Cre^* mice. There was a significant increase in left ventricular hypertrophy at 9 months, which led to an increase in expression of fetal genes, patches of fibrosis, increase in left ventricular mass, and reduced cardiac function from 10 months — all of which recapitulate features of the sarcomeric phenotype of HCM. Therefore, the developmental origin of HCM in *ROCKDN^Gata5-Cre^* mice is sarcomeric disruption in embryonic cardiomyocytes, ultimately triggering pathological left ventricular hypertrophy and maladaptive cardiac remodeling and cardiac dysfunction.

The article "Disruption of embryonic ROCK signaling reproduces the sarcomeric phenotype of hypertrophic cardiomyopathy" was retracted in 2020. Reason: fabricated or falsified data.

## Version 1 03/05/2019

In-Press Preview

## Version 2 04/18/2019

Electronic publication
